This article has been retracted.

# Efficacy of Posterior Cervical Laminectomy and Decompression plus Lateral Mass Screw-Rod Internal Fixation in the Treatment of Multisegment Cervical Spinal Canal Stenosis and Effects on Cervical Curvature and Range of Motion Parameters

**DOI:** 10.1155/2021/6001877

**Published:** 2021-10-15

**Authors:** Bo Liu, Yufei Wang, Yaning Zhang

**Affiliations:** Linfen People's Hospital, Orthopedics Department, Linfen, Shanxi 041000, China

## Abstract

**Objective:**

To investigate the clinical effects of posterior laminectomy and decompression plus lateral mass screw-rod internal fixation for the treatment of multisegment cervical spinal canal stenosis and the improvement of cervical curvature and range of motion in patients.

**Methods:**

A total of 68 patients with multisegment cervical spinal stenosis who were treated in our hospital from January 2019 to June 2020 were selected and randomly divided into the control group and the observation group according to the random number table, with 34 patients in each group. The patients in the control group were treated with traditional posterior cervical open-door laminoplasty with silk suture fixation, while those in the observation group were treated with posterior cervical laminectomy and decompression plus lateral mass screw-rod internal fixation. The perioperative index of patients in the two groups was recorded, and the clinical efficacy of patients was evaluated. The patient's JOA score, cervical physiological curvature, and cervical range of motion were evaluated. The occurrence of complications was recorded during follow-up.

**Results:**

The amount of intraoperative bleeding and postoperative rehabilitation training time in the observation group was less than that in the control group (*P* < 0.05). There was no significant difference in operation time between the two groups (*P* > 0.05). The total effective rate of the observation group was significantly higher than that of the control group (*P* < 0.05). The JOA scores at 1 week, 6 months, and 12 months after operation in the observation group were higher than those in the control group (*P* < 0.05). The physiological curvature of cervical spine in the observation group at 1 week, 6 months, and 12 months after operation was higher than that in the control group (*P* < 0.05). The cervical range of motion at 12 months after operation in the observation group was significantly higher than that in the control group (*P* < 0.05). The incidence of postoperative complications in patients of the observation group was significantly lower than that of the control group (*P* < 0.05).

**Conclusion:**

Posterior laminectomy and decompression plus lateral mass screw-rod internal fixation can help patients to improve various clinical symptoms caused by nerve compression and obtain better improvement of cervical curvature and range of motion. It is an ideal surgical method for the treatment of multisegment cervical spinal canal stenosis, and it is conducive to improving the clinical efficacy of patients.

## 1. Introduction

Cervical spondylotic myelopathy is a common and frequently occurring disease in orthopedics clinics, and cervical spinal stenosis is one of the important pathological bases of cervical spondylotic myelopathy [1, 2]. Multisegment cervical spinal canal stenosis is a severe cervical degenerative disease, which is mainly caused by factors such as ossification of the posterior longitudinal ligament of the cervical spine, multisegment cervical disc herniation, hypertrophy of ligamentum flavum, hyperplasia of articular processes, and developmental cervical spinal canal stenosis, thus causing blood circulation disorders of the spinal cord, compression of nerve roots and spinal cord, and finally the corresponding nerve root and spinal cord symptoms [3, 4]. Patients with multisegment cervical spinal canal stenosis are in severe condition and have high disability rate. Clinically, once patients have symptoms of spinal cord compression, surgery is the main treatment, but there is no uniform surgical standard, and different surgical methods have different effects. For multilevel cervical spinal stenosis, because the anterior approach surgery cannot directly remove the compression-causing substances in the spinal cord, and has many complications and poor long-term effect, posterior treatment is often advocated, which is mainly based on hemilaminectomy or total laminectomy and decompression laminoplasty. It can enlarge the volume of the spinal canal and achieve the purpose of decompression, but it cannot excessively destroy the stability of the cervical vertebra [5, 6]. In the traditional single-door surgery for posterior approach to neck, bone blocks and suture techniques are mainly used for the fixation of the vertebral plate on the portal axis side, in which the spinal process is sutured on the tough small joint capsule on the opposite side, so as to maintain the continuous opening of the spinal canal on the portal side. However, there is the problem of incomplete decompression on the hinge side, and suture tension or fracture may lead to the risk of lamina invagination after operation, with many complications [7, 8]. Therefore, the traditional single-door surgery has certain limitations. Posterior cervical laminectomy and decompression plus lateral mass nail-rod internal fixation, in which the lateral mass nail rod was specially added as the internal fixation material, exhibited good biocompatibility and high strength and toughness, thus meeting the structural requirements of human laminae [9–12]. Posterior cervical laminectomy and decompression plus lateral mass screw-rod internal fixation have a wide range of indications, which are mainly used in (1) those in the stage of spinal cord compression ≥3; (2) the ossification of the longitudinal ligament behind cervical vertebra suffers from spinal cord compression, which is difficult to be decompressed through anterior approach surgery; (3) the compression of cervical spinal cord comes from the calcification or hypertrophy of yellow ligament at the rear; (4) patients still having symptoms of spinal cord compression after anterior surgery; (5) patients who had anterior-posterior compression of the cervical spinal cord and the absolute value of the anterior-posterior diameter of spinal canal <10 mm. In this study, we compared the therapeutic effects of traditional posterior cervical open-door laminoplasty with silk suture fixation and posterior cervical laminectomy plus lateral mass screw-rod internal fixation, in order to provide reference for the clinical treatment of patients with multisegment cervical spinal canal stenosis.

## 2. Data and Methods

### 2.1. General Information

A total of 68 patients with multisegment cervical spinal stenosis were selected from January 2019 to June 2020 in our hospital, including 46 males and 22 females, with the average age of 61.73 ± 5.12 years and the average course of disease of 2.98 ± 0.51 years. Lesion segments: C_3–5_, 31 patients, and C_3–6_, 37 patients. The anterior-posterior diameter of the dural sac was (2.90 ± 1.39) mm, and the spinal cord drift was (4.50 ± 1.15) mm. The patients were divided into the control group (*n* = 34) and the observation group (*n* = 34) according to the random number table. The patients in the control group were treated with traditional posterior cervical open-door laminoplasty with silk suture fixation, while those in the observation group were treated with posterior cervical laminectomy and decompression plus lateral mass screw-rod internal fixation. This study was approved by the Hospital Ethics Committee, and informed consent was obtained from all patients and their families.

### 2.2. Inclusion Criteria

1. Presurgery diagnosis is confirmed through imaging examinations (X-ray, CT, and MRI). The number of vertebral segments is 3 or more.
2. After 6 months of conservative treatment, it is ineffective.
3. There are symptoms of spinal cord compression in different degrees.

### 2.3. Exclusion Criteria

1. Complicated with severe diseases of heart, brain, and other important organs.
2. Chronic diseases such as hypertension and diabetes are not stably controlled.
3. Patients complicated with space-occupying lesion in cervical spinal canal, fracture and dislocation of cervical vertebra, tumor of cervical vertebra, and severe instability.
4. Patients who failed to follow doctor's advice, withdrew from the study midway, or had incomplete follow-up information.

### 2.4. Research Methods

In the control group, the patients were treated with the traditional unilateral open-door laminoplasty with silk suture fixation via posterior approach. The patients were under general anesthesia with tracheal intubation, and the rats were placed on a stand-alone head rest bracket bed in the prone position, with the neck kept in a mild flexion position, and an incision was made in the middle of the posterior neck. The vertebral body position was confirmed by fluoroscopic examination with a C-arm X-ray machine, and the bilateral vertebral plates were fully exposed. The base of the spinous process was selected for drilling, and the edge of the outer edge of vertebral plate was selected for bone groove opening. The side with severe symptoms was taken as the door opening side, and the side with milder symptoms was taken as the hinge side. After the complete incision was made, a lead wire was punched in spinous process and sutured to the attachment point of the articular capsule tendon. The suture was retained, and the vertebral plate was lifted for 10 mm to open the door at a 30 angle. The incision was fully rinsed with normal saline to stop bleeding and suture the incision.

In the observation group, posterior cervical laminectomy and decompression plus lateral mass nail-rod internal fixation was adopted. The patients were under general anesthesia with intubation, and they were placed on a stand-alone head rest bracket bed in the prone position. The neck was kept in a mild flexion position, and an incision was made in the middle of the cervical back. The skin, subcutaneous, and fascia were cut layer by layer, and the bilateral paravertebral muscles were peeled open to expose spinous process, bilateral laminae, and lateral mass. The side with more severe symptoms was selected as the door opening side. The needle insertion point and angle were determined according to Magerl technique. The lateral mass screw was inserted after sounding. After the screw position was confirmed to be good by fluoroscopy with C-arm X-ray machine, posterior resection of the posterior wall of the spinal canal at the corresponding segment was performed, paying attention to the protection of the lateral mass bone. The vertebral plate was completely removed by using thin bone-biting forceps to completely decompress the spinal canal. After traction by contact cranial ring arch, prebent titanium rod was linked to the screw, and the screw was fixed by screwing the rod for orthopedic purposes. The spinous process and the lamina bone substance after the bite were trimmed into fine particles for bone grafting between the bilateral small customs. A negative pressure drainage tube was placed and sutured layer by layer. According to the drainage condition, they were removed 48–72 hours after operation. After the catheter was removed, the patient was guided to perform functional exercise under the protection of the neck brace.

### 2.5. Observation Indicators

The data of gender, age, course of disease, and clinical manifestation were collected and compared between the two groups. The intraoperative bleeding volume, operation time, and postoperative rehabilitation training time were recorded in the two groups.

To evaluate the clinical efficacy of patients. (1) Marked effectiveness: after treatment, the symptoms of spinal compression completely disappeared, and the curvature of cervical spine returned to the normal level, so the patient could move freely. (2) Effectiveness: after treatment, the symptoms of spinal compression were obviously improved, and the curvature of cervical spine was reduced as compared with that before treatment. However, the range of motion was limited to a certain extent. (3) Invalid: after treatment, the symptoms improved slightly, the curvature of cervical vertebra did not change obviously, and the range of motion was limited.

The JOA score and the physiological curvature of the cervical spine (the angle between the C2 lower endplate and the C7 lower endplate on the cervical lateral X-ray) were evaluated 1 week after operation and 6 or 12 months after operation, respectively. The cervical range of motion (the angle between the C2 lower endplate and the C7 lower endplate on the cervical hyperextension and hyperflexion radiography) was compared postoperatively and at the end of the follow-up. Complications were recorded during the follow-up.

### 2.6. Statistical Methods

The results of this experiment were statistically analyzed by SPSS 20.0 (SPSS Co. Ltd., Chicago, USA). Count data were expressed by rate, and chi-square test was used for their comparison between groups. Measurement data were expressed by mean ± standard deviation, the analysis of variance using repeated measurement design was compared, and *t*-test was used for their comparison between groups. *P* < 0.05 indicates that the difference is statistically significant.

## 3. Results

### 3.1. Comparison of the General Data between Two Groups

There was no significant difference between two groups in gender, age, course of disease, limb numbness, limb pain, lower limb walking weakness, chest and abdomen banding feeling, positive Hoffmann sign, and other clinical manifestations (*P* > 0.05) as shown in Table 1.

### 3.2. Comparison of Surgical Condition and Postoperative Rehabilitation Training Time between Two Groups

The amount of intraoperative bleeding and postoperative rehabilitation training time in the observation group was less than that in the control group, and the difference was statistically significant (*P* < 0.05). There was no significant difference in the operation time between the two groups (*P* > 0.05) as shown in Figure 1.

### 3.3. Comparison of Clinical Efficacy between Two Groups

The total effective rate of the observation group was significantly higher than that of the control group (*P* < 0.05) as shown in Figure 2.

### 3.4. Comparison of JOA Scores between Two Groups

The JOA scores were improved in all patients after operation. The JOA scores at 1 week, 6 months and 12 months after operation in the observation group were higher than those in the control group, and the differences were statistically significant (*P* < 0.05). As show in Figure 3.

### 3.5. Comparison of Cervical Physiological Curvature between Two Group

The physiological curvature of cervical spine was improved in all patients after operation. The physiological curvature of cervical spine in the observation group at 1 week, 6 months, and 12 months after operation was higher than that in the control group, and the difference was statistically significant (*P* < 0.05) as shown in Figure 4.

### 3.6. Comparison of Cervical Range of Motion between Two Groups

The cervical range of motion was improved in all patients after operation. The cervical range of motion at 12 months after operation in the observation group was significantly higher than that in the control group, and the difference was statistically significant (*P* < 0.05) as shown in Figure 5.

### 3.7. Comparison of Postoperative Complications between Two Groups

The incidence of postoperative complications in patients of the observation group was significantly lower than that of the control group, and the difference was statistically significant (*P* < 0.05) as shown in Figure 6.

## 4. Discussion

The cervical semispinous muscle is an important dynamic stabilizing factor for maintaining the normal sagittal sequence [13, 14]. The maintenance of the normal sequence of the cervical vertebrae after posterior surgery mainly depends on the dynamic systems such as muscles and ligaments, rather than osseous fusion or other rigid structures [15, 16]. The amount of intraoperative bleeding and postoperative rehabilitation training time in the observation group were significantly lower than those in the control group. This is because the decompression range is flexibly controlled by posterior cervical laminectomy and lateral mass nail and rod fixation, which makes the operation easier and the incision smaller than the traditional operation, thus reducing the amount of intraoperative bleeding and postoperative infection rate. Compared with traditional surgical methods, the excellent rate and good healing rate of the surgical incision is also significantly improved, and the time of postoperative rehabilitation training was significantly shortened. The study showed that the total effective rate of the observation group reached 97.06%, significantly higher than that of the control group. Posterior laminectomy and decompression combined with lateral mass screw-rod internal fixation can maintain the stability of cervical vertebra after operation in time, maintain an effective physiological curvature of the cervical vertebra, and reduce the incidence of cervical instability or even kyphosis after operation [17].

The operation process of postoperative double disc surgery was summarized, and the operation skills and precautions were summarized. It was considered that, before surgery in the prone position, the use of wide tape to tighten the skin of bilateral shoulders and back of the patient was conducive for better exposure of the surgical field of view during the operation. When the bilateral paravertebral muscles of the patient are separated by surgery, the electrotome should be operated slowly and gently, so as to reduce intraoperative bleeding as much as possible. Under the condition of completely protecting the lamina, the lateral mass screws were positioned and placed, and the residual cortical bone was removed with a thin cervical plate chisel. When the dura mater adheres to the lamina or ligamentum flavum, laminectomy should be performed after careful separation, so as to prevent the dura mater from being damaged or torn, resulting in spinal cord injury. If epidural injury occurs during the operation, the surface of the dura will be covered with biofilm patch or gelatin sponge, and the drainage tube will be placed for postoperative drainage.

Posterior cervical laminectomy and decompression combined with lateral mass screw and rod fixation is developed on the basis of traditional posterior single-door operation. The main points of the operation are to expand the spinal canal during the operation, keep the spinal canal expanded after the operation, and prevent restenosis, so as to indirectly relieve the compression of the anterior part of the spinal cord, realizing the treatment of cervical spinal stenosis, and improving the microcirculation perfusion of the patient's spinal cord [18]. In this study, the JOA score, cervical physiological curvature, and cervical range of motion were recorded during the follow-up visit. The results showed that the JOA score, cervical physiological curvature, and cervical range of motion in the observation group were better than those in the control group. The accuracy and reliability of the operation were verified.

Postoperative chronic pain and C5 nerve root palsy are common complications of traditional posterior cervical approach, and their clinical incidence is high, which seriously affects the normal life of patients [19, 20]. The incidence of postoperative complications in patients of the observation group was significantly lower than that of the control group. Compared with the traditional posterior cervical single-door expanded plastic suture fixation, posterior cervical laminectomy and decompression combined with lateral mass nail and rod internal fixation can fix the cervical spine immediately, promote cervical bone grafting and fusion, maintain the physiological curvature of cervical spine, prevent long-term deformity, and achieve better initial stability of the cervical spine after operation. During the follow-up, no loosening or displacement of internal fixation was found, and the cervical spine maintained a good physiological curvature. It is proved that the lateral mass nail-rod system is reliable and does not affect spinal cord decompression, which is a good method for posterior cervical fixation [21].

Posterior cervical laminectomy and decompression plus lateral mass screw-rod internal fixation can help patients to improve various clinical symptoms caused by nerve compression and obtain better improvement of cervical curvature and range of motion. It is an ideal surgical method for the treatment of multisegment cervical spinal canal stenosis and helps to improve the clinical efficacy of patients.

## Figures and Tables

**Figure 1:** Comparison of surgical condition and postoperative rehabilitation training time between two groups. Note: compared with the control group, ^*∗*^*P* < 0.05.

**Figure 2:** Comparison of clinical efficacy between two groups. Note: compared with the control group, ^*∗*^*P* < 0.05.

**Figure 3:** Comparison of JOA scores between two groups. Note: compared with the control group, ^*∗*^*P* < 0.05.

**Figure 4:** Comparison of cervical physiological curvature between two groups. Note: compared with the control group, ^*∗*^*P* < 0.05.

**Figure 5:** Comparison of cervical range of motion between two groups. Note: compared with the control group, ^*∗*^*P* < 0.05.

**Figure 6:** Comparison of postoperative complications between two groups. Note: compared with the control group, ^*∗*^*P* < 0.05.

**Table 1:** Comparison of the general data between two groups.

Project		Control group (*n* = 34)	Observation group (*n* = 34)	*t*/*χ*^*2*^ value	*P* value
Gender	Male	22	24	0.269	0.604
	Female	12	10		
Age (years)		61.05 ± 5.16	62.71 ± 5.52	1.281	0.205
Course of disease (years)		2.94 ± 0.53	3.02 ± 0.49	0.646	0.520
Clinical symptoms	Numbness of limbs	31	29	0.567	0.452
	Limb pain	28	26	0.360	0.549
	Walking weakness of lower limbs	25	27	0.327	0.567
	Belted chest and abdomen	19	20	0.060	0.806
	Hoffmann's sign being positive	32	30	0.731	0.393

## Data Availability

The data can be obtained from the author upon reasonable request.
